# Improvement of Student Weariness Emotion in English Classroom Based on Intelligent Internet of Things and Big Data Technology

**DOI:** 10.1155/2022/9369389

**Published:** 2022-08-31

**Authors:** Ya Pang

**Affiliations:** School of Foreign Languages, Hainan Normal University, Haikou, Hainan 571158, China

## Abstract

In order to improve the recognition effect of student weariness emotion in English classroom, this paper combines intelligent Internet of Things technology and big data technology to construct an improvement model of student weariness emotion in English classroom. In the process of student facial expression recognition, according to the given grayscale threshold, this paper extracts the surface contour information from the three-dimensional volume data, extracts the student's surface contour information, and uses triangular facets to fit to form a triangular mesh. Moreover, this paper renders a triangular mesh model and shows how to speed up the calculation of PFH. In addition, this paper proposes a Fast Point Feature Histogram, which uses an iterative closest point fine registration algorithm for image registration. Finally, this paper constructs an emotion recognition model of students' weariness in English classroom. From the test results, it can be seen that the student weariness emotion recognition system in English classroom proposed in this paper can effectively identify students' weariness emotion.

## 1. Introduction

Social development is very important to the growth of young people, and the wide application of the Internet has a subtle influence on the physical and mental health of young people. It can be seen that promoting the mental health of adolescents requires the coordinated maintenance of families, schools, society, and the Internet. Cognitive therapy has proved through a series of studies that painful and negative cognition is the main feature of psychological problems [1]. The focus of family, school, social, and network interventions is to transform students' and parents' automatic thinking and cognition of intermediate beliefs or core beliefs, and to find a method suitable for the student's specific situation is the most critical [2]. Judging from the reactions of parents, the main family conflicts are caused by children's procrastination and dislike of school, but there are hidden reasons such as parent-child relationship problems caused by parent-child communication and improper parenting methods [3], in particular parents' unreasonable understanding and interpretation of their children's problem behaviors. The specific reasons are analyzed as follows. The first reason is family and social life, such as the absence of a father. After the divorce, the mother had no time to take care of the child due to her busy work, and her grandparents picked up the child to take care of the child's food and daily life. At this time, because grandparents dote on their children, they often follow their children to meet their demands. The second reason is family education [4]. Since parents focus on their children's academic performance, they ignore their children's psychological needs. Moreover, they have not established a clear sense of rules for their children since childhood, and the family's parenting method is not applicable and does not match the child's situation. The third reason is the aspect of personal cognitive conflict. The normal adaptive behavior and personality characteristics of children are given negative explanations such as procrastination and introversion by parents. At the same time, parents use urging, criticism, reasoning, and other methods to imply and reinforce such views, so that children have core beliefs such as “I'm not good enough” and “I'm not worthy of love,” causing them to resist parents. Moreover, the expectations of both parties are inconsistent, the cognitive model of weariness is caused by distorted and biased thinking styles, and the individual is adversely affected by his negative thoughts about self, experience, and future [5].

The questionnaire shows that more than 85% of the students have different degrees of weariness. Most students who are tired of learning know the importance of learning, but they cannot control themselves. According to the degree of student weariness, it can be divided into general weariness and weariness. General dislike of learning is mainly a negative emotion common to learning. The main manifestations are often complaining about being very tired from studying, having thoughts of unwillingness to study, deserting in class, occasionally failing to complete homework, and skipping classes. Such school weariness and behavior are generally transient, and students can overcome it through self-adjustment, which generally does not affect normal learning [6]. The main manifestations of school weariness are that there is a big deviation in students' understanding of learning, and their emotions are particularly disgusting to study, and students take the initiative to stay away from learning. Such students often lose interest and confidence in learning because of unclear learning goals, regard learning as a burden, lack desire for knowledge, dislike homework, and fear exams and are just forced and mechanically coping with learning [7]. Such students often do not pay attention to class, do not complete homework, often sleep in class or violate class discipline, skip classes, and even drop out of school. More serious psychological symptoms such as headaches and stomach pains will appear, and they will not be able to study normally [8].

Learning weariness is a psychological state in which students are extremely disgusted with learning activities. Its explicit features are truancy, not doing homework, disagreeing with teachers and classmates in class, and failing to abide by school-level school rules in school. The concrete manifestation of life dissatisfaction seriously affects the daily learning order of the school and reduces students' enthusiasm for learning [9]. Scholars at home and abroad have put forward different views on students' weariness. In the process of learning, students' self-efficacy is too low, unable to obtain a sense of satisfaction and achievement, and their grades are not satisfactory, so they gradually lose interest in learning, resulting in the psychological weariness of learning [10]. Students' failure to obtain the expected results through hard work and the loss of confidence in their study and life because of the tense employment situation are the main reasons for students' weariness [11]. Scholars generally attribute the problem of students' weariness to students' sense of failure from childhood rather than achievement, parents and teachers' incomprehension, fear of being scolded, and students' failure to master the correct and suitable learning methods. Cheng et al. believe that failure to develop good study habits and ideological resistance to study are the main reasons for college students to be tired of learning [12]. There are three psychological attributions to students' dislike of learning: (1) students who have poor academic performance, have cognitive deviations in learning functions, think that efforts are useless and do not want to work hard, and are in a state of numbness to learning. They think that studying is a waste of time and even have extreme ideas such as “the more you study, the less your income” and “the higher the diploma, the lower the salary.” The current increasingly tense employment environment and pressure make them feel that a diploma is worthwhile. The level is not proportional to the future employment and income, so they have disgust and dissatisfaction with the school life, so they do not cooperate in class or even miss class and do not complete homework after class [13]. (2) There is a cognitive bias towards learning attitudes, a very low sense of self-efficacy, and there is no joy in learning, so there is a feeling of resistance to learning activities. Students at the vocational stage are in their adolescence, and they lack stamina to do things and are easily attracted by new things from the outside world. However, due to the constant pressure from parents and teachers, they have to study step by step. However, in the process of learning activities, most of them have negative emotions such as anxiety, irritability, anxiety, and fear. They have not really experienced the sense of achievement and happiness brought by active learning, so they hate going to school, are afraid of teachers, and resist completing homework [14]. (3) In a state of passive learning for a long time, there is a cognitive bias in learning activities, and learning is a burden. Vocational students are still in their adolescence, and they are prone to rebellious psychology. They think that the mainstream activity of learning is not suitable for them. Ji, even running away from home or dropping out of school, has long been in opposition to teachers and parents and is unwilling to open up their inner world with their elders [15].

Scholars often study the influencing factors of orientation/weariness from the perspective of “weariness.” Literature [16], from the perspective of educational culture, believes that the loss of free, independent, and critical university spirit is the deep-seated incentive for college students to be disgusted with learning. From the perspective of educational psychology, some scholars have studied the phenomenon of college students' orientation/weariness. By establishing a structural equation model, it is concluded that core self-evaluation has direct and indirect effects on college students' weariness. The conclusion is that there is a mediating effect on the influence of college students' weariness [17]. Studies have shown that learning weariness is significantly correlated with learning burnout, core self-evaluation, and professional commitment [18]. This type of research involves the influence of school education system, teaching method, school education purpose, and school curriculum on learning orientation/weariness [19]. By classifying learning motivation, living arrangements, and personal planning as personal factors that affect learning/aversion to learning and classifying social value, teacher charisma, and curriculum as environmental factors, it is concluded that the other five factors other than curriculum can predict college students. The unsatisfactory college environment has a negative effect on college students' learning [20].

This paper combines intelligent Internet of Things technology and big data technology to construct an improvement model for students' weariness in English classrooms and promote the construction of mental health of college English classroom students.

## 2. Student's Facial Weariness Emotion Recognition Algorithm

The algorithm involves the concept of “isosurface” (surface contour). The reason is that the algorithm is based on surface rendering, which treats two-dimensional slice data as a three-dimensional data system, such as the eight vertices of two adjacent slices as cube data. Then, according to a given grayscale threshold, the surface contour information is extracted from the three-dimensional volume data, so the algorithm is also called “isosurface extraction method.” In the three-dimensional voxel space, the isosurface can be represented as a set of pixel points with the same gray value, which can be represented by

(1) $$\begin{array}{c} \left\{\left(x,y,z\right),f\left(x,y,z\right)=c_{0}\right\}. \end{array}$$

After the refined CAD model and the reconstructed model of the student's facial expression image are discretized into a point cloud, the three-dimensional coordinate information of the model is available. When this information is obtained, registration can be performed. The process of performing registration is actually a process of unifying the measurement coordinate system of the model to be registered and the design coordinate system of the CAD model through rotation and translation transformation (such as rigid body transformation). In the three-dimensional coordinate system, people stipulate that the right-handed helical direction is the positive direction of the rotation transformation, that is, the clockwise direction from the origin to the positive half-axis of a certain coordinate axis. The basic rotation and translation transformations involved in rigid body transformation are as follows:

(2) $$\begin{array}{c} R\left(X,\alpha \right)=\left(\begin{array}{ccc} 1 & 0 & 0\\ 0 & \cos\alpha & \sin\alpha \\ 0 & -\sin\alpha & \cos\alpha \end{array}\right), \end{array}$$

(3) $$\begin{array}{c} R\left(Y,\beta \right)=\left(\begin{array}{ccc} \cos\beta & 0 & -\sin\beta \\ 0 & 1 & 0\\ \text{sn}\beta & 0 & \cos\beta \end{array}\right), \end{array}$$

(4) $$\begin{array}{c} R\left(Z,\gamma \right)=\left(\begin{array}{ccc} \cos\gamma & \sin\gamma & 0\\ -\sin\gamma & \cos\gamma & 0\\ 0 & 0 & 1 \end{array}\right). \end{array}$$

*R*(*X*, *α*) represents a rotation around the *x*-axis, *R*(*Y*, *β*) represents a rotation around the *y*-axis *β*, and *R*(*Z*, *γ*) represents a rotation of *Y* around the *z-*axis. Then, the rotation transformation matrix *R*_3×*x*_ in three-dimensional space can be expressed as follows:

(5) $$\begin{array}{c} R_{3\times x}=R\left(X,\alpha \right),R\left(Y,\beta \right),R\left(Z,\gamma \right)=\left(\begin{array}{ccc} 1 & 0 & 0\\ 0 & \cos\alpha & \sin\alpha \\ 0 & -\sin\alpha & \cos\alpha \end{array}\right)\left(\begin{array}{ccc} \cos\beta & 0 & -\sin\beta \\ 0 & 1 & 0\\ \sin\beta & 0 & \cos\beta \end{array}\right)\left(\begin{array}{ccc} \cos\gamma & \sin\gamma & 0\\ -\sin\gamma & \cos\gamma & 0\\ 0 & 0 & 1 \end{array}\right)=\left(\begin{array}{ccc} \cos\beta \cos\gamma & \cos\beta \sin\gamma & -\sin\beta \\ -\cos\alpha \cos\gamma -\sin\alpha \sin\beta \cos\gamma & \cos\alpha \cos\gamma +\sin\alpha \sin\beta \cos\gamma & \sin\alpha \cos\beta \\ \sin\alpha \sin\gamma +\cos\alpha \sin\beta \cos\gamma & -\sin\alpha \cos\gamma -\cos\alpha \sin\beta \sin\gamma & \cos\alpha \cos\beta \end{array}\right). \end{array}$$

The basic principle of point cloud registration is to transform the point cloud to be registered to the target point cloud through rotation and translation transformation (rigid body transformation). At this time, the coordinate systems of the two point clouds are unified, and the three-dimensional space rigid body transformation *T* is as follows:

(6) $$\begin{array}{c} T:\left(\begin{array}{c} x^{\prime }\\ y^{\prime }\\ z^{\prime } \end{array}\right)=R\left(\begin{array}{c} x\\ y\\ z \end{array}\right)+\left(\begin{array}{c} t_{x}\\ t_{y}\\ t_{z} \end{array}\right). \end{array}$$

Among them, *t*_*x*_, *t*_*x*_, and *t*_*z*_ describe the translation in each direction of *X*, *Y*, and *Z*, respectively, and *θ* represents the rotation angle between the two point clouds.

At present, most of the fine registration techniques use the iterative closest point (ICP) algorithm. The premise of using this algorithm is that it needs to have a good initial alignment posture, so the initial registration method has to be used to initially align the object to be registered and the design model. There are many initial registration methods at this stage, but the common purpose is to create a good initial condition for fine registration.

At present, there are many initial registration methods, and specific problems should be analyzed in detail when selecting them. If the experimental object is a relatively complete three-dimensional model, an initial registration method based on global features, such as a covariance matrix- (CDB-) based initial registration method, should be used. On the contrary, if the experimental object is a three-dimensional model reconstructed from incomplete data, an initial registration method based on local features, such as the normal distribution transformation (NDT) initial registration method, should be used. The initial registration methods involved in this paper include registration method based on covariance matrix (CDB), initial registration method based on normal distribution transform (NDT), and registration method based on sampling consistency initial alignment (SAC-IA).

The first is the initial registration based on the covariance matrix. As the name suggests, this method needs to calculate the covariance matrix. Its basic idea is similar to principal component analysis (PCA), which is a dimensionality reduction algorithm based on global features. Its principle diagram is as shown in Figure 1.

As shown in Figure 1, the coordinate system XOy is the world coordinate system, and the principal component analysis is performed on the scattered points in the figure, and the coordinate system uOv can be obtained through the coordinate rotation transformation obtained by calculation, which is the main axis coordinate system. Moreover, each scatter point is projected onto the main axis coordinate system 1Ov and the world coordinate system XOy, the information is better preserved, and the dimension of the analysis is reduced.

Formula (7) is used to calculate the covariance matrix of the point cloud image:

(7) $$\begin{array}{c} \text{Cov}=\frac{1}{N}\overset{N-1}{\underset{i=0}{\sum }}\left(p_{i}-\bar{p}\right){\left(p_{i}-\bar{p}\right)}^{T}. \end{array}$$

Among them, *N* is the total number of points in the point cloud image, *p* is the center of the point cloud, and *p*_*i*_ is the *i*-th point on the surface of the point cloud.

It can be obtained by the similar diagonalization:

(8) $$\begin{array}{c} {\text{Cov}}_{k}=U_{k}D_{k}U_{k}^{T}. \end{array}$$

Among them, *k* = 1, 2 represents the target point cloud and the point cloud to be registered, *t*_*x*_ is a diagonal matrix composed of eigenvalues, and *U*_*k*_ is a matrix composed of eigenvectors in the principal axis direction.

The rotation matrix is shown in

(9) $$\begin{array}{c} R=U_{1}U_{2}^{-1}. \end{array}$$

The translation vector *t* is determined by the centroids of the two point clouds, as shown in

(10) $$\begin{array}{c} t={\bar{\mu }}_{1}-R{\bar{\mu }}_{2}. \end{array}$$

The second method of initial registration is the normal distribution transform (NDT) initial registration algorithm. This method is actually an extended application of the registration method based on the covariance matrix. The difference is that NDT does not compare the point-to-point distance between the point cloud of the entire CT image surface reconstruction model and the point cloud of the CAD model. Instead, the point cloud of the CAD model is first processed into blocks and then converted into a normal distribution of multidimensional variables as a reference system. If the rigid body transformation parameters can make the CT image surface reconstruction model point cloud match the CAD model point cloud well, then the probability density of the CT image surface reconstruction model point cloud in the reference frame will be larger. Therefore, it is an initial registration method based on local features.

The probability density function of the random variables involved is as follows:

(11) $$\begin{array}{c} f\left(x\right)=\frac{1}{\sigma \sqrt{\left(2\pi \right)}}e^{-\left(\left({\left(x-\bar{\mu }\right)}^{2}\right)/2\sigma^{2}\right)}. \end{array}$$

The probability density function of a random vector is

(12) $$\begin{array}{c} f\left(x\right)=\frac{1}{{\left(2\pi \right)}^{D/2}\sqrt{\sum }}e^{-\left(\left({\left(x-\bar{\mu }\right)}^{T}\overset{-1}{\sum }\left(x-\bar{\mu }\right)\right)/2\sigma^{2}\right)}. \end{array}$$

When using the normal distribution to represent discrete point clouds, each probability density function can be viewed as an approximation of a local surface because each patch is continuously differentiable. It expresses a lot of information about the surface, such as curvature and orientation.

In the process of using the normal distribution transform (NDT) for initial registration, the most commonly used method is Newton's method when it comes to solving the optimization problem. The basic principle of this method is to solve the root of the equation *f*(*x*) = 0 through the Taylor series of a certain function *f*(*x*). *f*(*x*) is expanded into a Taylor series at *x*:

(13) $$\begin{array}{c} f\left(x\right)=f\left(x_{0}\right)+f^{\prime }\left(x_{0}\right)\left(x-x_{0}\right)+\frac{1}{2}f^{\prime \prime }\left(x_{0}\right)\left(x-x_{0}\right)+.\cdots \end{array}$$

For convenience of example, the first-order part of equation (13) is considered here as an approximation of *f*(*x*). Therefore, the solution of *f*(*x*_0_) + *f*′(*x*_0_)(*x* − *x*_0_) = 0 can be regarded as an approximate solution of *f*(*x*) = 0, and the approximate solution is *x*_1_ = *x*_0_ − *f*(*x*_0_)/*f*′(*x*_0_). Because here it is only a linear expansion of the Taylor series of *f*(*x*), so *x* is not a solution of *f*(*x*) = 0, and it is just an approximate solution, but it can be said that *f*(*x*_1_) is closer to zero than *f*(*x*_0_). If iterations are introduced, the resulting solution will be more precise, and *x*_*n*+1_ = *x*_*n*_ − *f*(*x*_*n*_)/*f*′(*x*_*n*_). The iterative process of solving the equation is shown in Figure 2.

From Figure 2, it can be clearly seen that each variable changes in the solution process, such as the previous value of *x* participates in the next iteration, that is, *x*_*k*+1_ = *x*_*k*_ − *f*(*x*_*k*_)/*f*′(*x*_*k*_), *x*_*k*_⟶*x*^∗^. *f*(*r*_*x*_) also approaches 0, that is, *f*(*x*_*k*_)⟶0. Thus, the solution *x*^∗^ of the equation *f*(*x*) = 0 is found.

The third is the sampling consistent initial alignment (SAC-IA) registration algorithm. Before mentioning this method, we have to point out an important concept: Point Feature Histogram (PFH). It obtains the histogram of the geometric information of the neighborhood around a center point by statistical methods and is a process of quantifying the difference in the neighborhood space around the center point. Its purpose is to map the average curvature of the surrounding neighborhood of a point as a geometric feature to a high-dimensional histogram, and multidimensional data has a lot of information that can express features. Specifically, the mapping of the feature histogram of a point is mainly based on the relationship between the point and the field of the point, and by calculating the relationship between the normals, the feature changes on the surface of the model are expressed. We can see that the normal of a point cloud is an extremely important feature.

As shown by the red point in Figure 3, this point is the center point of a sphere in a three-dimensional space. In the sphere, the center point and the *k* neighbor points around it are related to each other to form a “network.” The feature histogram of PFH is obtained by calculating the relationship between the center point and the surrounding neighborhood points.

We assume that there are two points *p*_1_ and *p*_2_ whose normal vectors are *n*_1_ and *n*_2_, respectively. Meanwhile, a three-dimensional local coordinate system is established at a certain point in it, and the unit vectors of the three-dimensional local coordinate system are *u*, *v*, and *w*. The creation rules of these vectors are as follows: *v* = *u* × (*p*_2_ − *p*_1_/‖*p*_2_ − *p*_1_‖_2_), *w* = *u* × *v*, *u* = *n*_1_. Among them, ‖*p*_2_ − *p*_1_‖_2_ represents the Euclidean distance between two points *p*_1_ and *p*_2_. After that, using the *uw* three-dimensional coordinate system described above, the difference between the normal vectors *n*_1_ and *n*_2_ can be represented by three angles (*e*, *g*, 0), and the establishment rules of the three angles are as follows: *α* = *v* · *n*_2_, *ϕ* = *u* · (*p*_2_ − *p*_1_/‖*p*_2_ − *p*_1_‖_2_), *θ*arctan(*w* · *n*_2_, *u* · *n*_2_). The three-dimensional local coordinate system of the two points is shown in Figure 4.

Afterwards, for the “point pair” formed by the center point in the sphere and its surrounding *k* neighborhoods, the local features can be mapped to the subintervals of the histogram as long as three angles <*α*, *p*, 0> are calculated. The original two points need 12 parameters (the coordinate information of each point and its normal and other parameters), but this new way of expressing features only needs to determine three parameters to contain all the information of the original two points.

In order to speed up the calculation of PFH, a Fast Point Feature Histogram (FPFH) I is proposed. This method adopts the means of simplification and optimization to speed up the calculation and can also seek the connection between different points in the point cloud. The formula of FPFH is as follows:

(14) $$\begin{array}{c} \text{FPFH}\left(p_{q}\right)=\text{SPFH}\left(p_{q}\right)+\frac{1}{k}\overset{k}{\underset{i=1}{\sum }}\frac{1}{w_{k}}\cdot \text{SPFH}\left(p_{k}\right). \end{array}$$

Among them, SPFH (Simplified Point Feature Histogram) in formula (14) is a simplified process of PFH. The algorithm consists only of querying the value of the (*α*, *ϕ*, *θ*) parameter for each center point. It is used to measure the distance between the center point and a certain neighborhood point , which can be called the weight of the point to*p*_*q*_ and a certain neighborhood point *p*_*k*_, which can be called the weight of the point to (*p*_*q*_, *p*_*k*_). The meaning of this weight is explained in Figure 5.

As shown in Figure 5, for the center point *p*_*q*_, the point and its neighbor points are connected with red line segments. It can be seen that the red line segment is the thickest, because these neighbor points are closest to the center point *p*_*q*_. It is not hard to see that the closer the two points are, the thicker the line segment connecting them. The FPFH algorithm first calculates the SPFH of the first center point and then uses the nearest neighbor point as the new center point to calculate the new SPFH. That is to say, combine the SPFH of the center point *p*_*q*_ itself with the SPFH of the neighbor point *p*. This update calculation can get the final FPFH of the more accurate center point *p*_*k*_. Compared with PFH, this FPFH method of weighted update calculation is more comprehensive and considers the correlation between neighborhoods. In short, the more times each point in the sphere is considered, the thicker the line segment representing the weight and the greater the impact on the center point.

The above is the theoretical knowledge involved in the three initial registration methods. With these theories, there are traces of which initial registration method to choose.

After performing the initial registration, the to-be-registered model can only be roughly aligned with the target model, so further fine registration needs to be performed. The most commonly used method for fine registration is the registration algorithm based on iterative closest point (ICP). However, this method is easy to fall into the state of local optimal solution, which makes the computer mistakenly think that the model has completed the registration, which is why the initial registration must be performed before the fine registration. In this paper, the iterative closest point fine registration algorithm is used without exception, and the algorithm is defined as follows:

If it is assumed that the source point cloud set *P* = {*p*_1_, *p*_2_, ⋯, *p*_*n*_} and the target point cloud set *Q* = {*q*_1_, *q*_2_, ⋯, *q*_*n*_} exist, the ICP fine registration algorithm obtains the corresponding transformation matrix (*R*, *t*) by minimizing the distance between the two points in the optimization theory:

(15) $$\begin{array}{c} \left(R,t\right)=\underset{R\in SO\left(d\right),t\in R^{d}}{\arg\min}\overset{n}{\underset{i=1}{\sum }}\omega_{i}\left\|\left({Rp}_{i}+t\right)-q_{i}\right\|. \end{array}$$

Among them, *ω*_*i*_ represents the weight of each point, *R* is the required rotation matrix, and *t* is the translation vector.

There are many ways to solve this equation. This paper introduces the method based on singular value decomposition (SVD), and the error function to be optimized by ICP fine registration is as follows:

(16) $$\begin{array}{c} F\left(R,t\right)=\overset{n}{\underset{i=1}{\sum }}\omega_{i}{\left\|\left({Rp}_{i}+t\right)-q_{i}\right\|}^{2}, \end{array}$$

(17) $$\begin{array}{c} f={\left\|\left({Rp}_{i}+t\right)-q_{i}\right\|}^{2}-{\left({Rp}_{i}+t-q_{i}\right)}^{T}\left({Rp}_{i}+t-q_{i}\right). \end{array}$$

First, the derivative with respect to *t* is computed and *df* is differentiated as

(18) $$\begin{array}{c} df=d\left({\left({Rp}_{i}+t-q_{i}\right)}^{T}\right)\left({Rp}_{i}+t-q_{i}\right)+{\left({Rp}_{i}+t-q_{i}\right)}^{T}d\left({Rp}_{i}+t-q_{i}\right)=\underset{d\left(X^{T}\right)={\left(dX\right)}^{T}}{\underbrace{{\left(\left({Rp}_{i}+t-q_{i}\right)\right)}^{T}}}\left({Rp}_{i}+t-q_{i}\right)+{\left({Rp}_{i}+t-q_{i}\right)}^{T}dt={\left(dt\right)}^{T}\left({Rp}_{i}+t-q_{i}\right)+{\left({Rp}_{i}+t-q_{i}\right)}^{T}dt=\underset{\text{when }A^{T}B\text{ is a scalar},A^{T}B=B^{T}A}{\underbrace{2{\left({Rp}_{i}+t-q_{i}\right)}^{T}dt}}. \end{array}$$

For *df* = (*∂f*^*T*^/*∂t*)*dt*, *∂f*/*∂t* = 2(*Rp*_*i*_ + *t* − *q*_*i*_) can be obtained in the same way. Therefore,

(19) $$\begin{array}{c} \frac{\partial F}{\partial t}=\overset{n}{\underset{i=1}{\sum }}2w_{i}\left({Rp}_{i}+t-q_{i}\right)=2t\overset{n}{\underset{i=1}{\sum }}w_{i}+2R\overset{n}{\underset{i=1}{\sum }}w_{i}p_{i}-2\overset{n}{\underset{i=1}{\sum }}w_{i}p_{i}. \end{array}$$

When *∂F*/*∂t* = 0, we can get

(20) $$\begin{array}{c} t=\frac{\sum_{i=1}^{n}w_{i}q_{i}-R\sum_{i=1}^{n}w_{i}p_{i}}{\sum_{i=1}^{n}w_{i}}. \end{array}$$

When $\bar{p}=\sum_{i=1}^{n}w_{i}p_{i}/\sum_{i=1}^{n}w_{i},\bar{q}=R\sum_{i=1}^{n}w_{i}q_{i}/\sum_{i=1}^{n}w_{i}$, formula (20) transforms into

(21) $$\begin{array}{c} t=\bar{q}-R\bar{p}. \end{array}$$

Substituting formula (21) into formula (16), we get

(22) $$\begin{array}{c} \overset{n}{\underset{i=1}{\sum }}\omega_{i}{\left\|\left({Rp}_{i}+t\right)-q_{i}\right\|}^{2}=\overset{n}{\underset{i=1}{\sum }}\omega_{i}{\left\|\left({Rp}_{i}+\bar{q}-R\bar{p}\right)-q_{i}\right\|}^{2}=\overset{n}{\underset{i=1}{\sum }}\omega_{i}{\left\|R\left(p_{i}-\bar{p}\right)-\left(p_{i}-\bar{q}\right)\right\|}^{2}. \end{array}$$

If , then the problem becomes

(23) $$\begin{array}{c} \left(R,t\right)=\underset{R\in SO\left(d\right)}{\arg\min}\overset{n}{\underset{i=1}{\sum }}\omega_{i}{\left\|{\text{Rx}}_{i}-y_{i}\right\|}^{2}. \end{array}$$

Next, the rotation matrix is computed by least squares:

(24) $$\begin{array}{c} {\left\|{\text{Rx}}_{i}-y_{i}\right\|}^{2}={\left({\text{Rx}}_{i}-y_{i}\right)}^{T}\;\left({\text{Rx}}_{i}-y_{i}\right)=\left({x_{i}}^{T}R^{T}-{y_{i}}^{T}\right)\;\left({\text{Rx}}_{i}-y_{i}\right)=\underset{R\text{ is the unit of orthogonal array},{RR}^{T}=1}{\underbrace{{x_{i}}^{T}R^{T}{\text{Rx}}_{i}}}-{y_{i}}^{T}{\text{Rx}}_{i}-{x_{i}}^{T}R^{T}y_{i}+{y_{i}}^{T}\;y_{i}={x_{i}}^{T}x_{i}-{y_{i}}^{T}{\text{Rx}}_{i}-\underset{{\left(\text{AB}\right)}^{T}=B^{T}A^{T}}{\underbrace{{\left({\text{Rx}}_{i}\right)}^{T}y_{i}}}+{y_{i}}^{T}\;y_{i}={x_{i}}^{T}x_{i}-\underset{\text{when }A^{T}B\text{ is a scalar},A^{T}B=B^{T}A}{\underbrace{2{y_{i}}^{T}{\text{Rx}}_{i}}}+{y_{i}}^{T}y_{i}. \end{array}$$

The final question turns into

(25) $$\begin{array}{c} \underset{R\in \text{SO}\left(d\right)}{\arg\min}\overset{n}{\underset{i=1}{\sum }}w_{i}{\left\|{\text{Rx}}_{i}-y_{i}\right\|}^{2}=\underset{R\in \text{SO}\left(d\right)}{\arg\min}\overset{n}{\underset{i=1}{\sum }}w_{i}\underset{x_{i},y_{i}\text{ is independent of }R}{\underbrace{\left({x_{i}}^{T}x_{i}-2{y_{i}}^{T}{\text{Rx}}_{i}+{y_{i}}^{T}y_{i}\right)}}=\underset{R\in \text{SO}\left(d\right)}{\arg\min}\overset{n}{\underset{i=1}{\sum }}w_{i}{y_{i}}^{T}{\text{Rx}}_{i}. \end{array}$$

Then, there is

(26) $$\begin{array}{c} W_{n\times n}Y_{n\times 3}^{T}R_{3\times 3}X_{3\times n}=\left[\begin{array}{cccc} w_{1} & \; & \; & \;\\ \; & w_{2} & \; & \;\\ \; & \; & \ddots & \;\\ \; & \; & \; & w_{n} \end{array}\right]\left[\begin{array}{c} -y_{1}^{T}-\\ -y_{2}^{T}-\\ \vdots \\ -y_{n}^{T}- \end{array}\right]\left[\begin{array}{c} \;\\ R\\ \; \end{array}\right]\left[\begin{array}{ccc} \left|\;\right. & \left|\;\right. & \left|\;\right.\\ x_{1} & x_{2}\cdots & x_{n}\\ \left|\;\right. & \left|\;\right. & \left|\;\right. \end{array}\right]=\left[\begin{array}{c} -w_{1}y_{1}^{T}-\\ -w_{2}y_{2}^{T}-\\ \vdots \\ -w_{n}y_{n}^{T}- \end{array}\right]{\left[\begin{array}{ccc} \left|\;\right. & \left|\;\right. & \left|\;\right.\\ {\text{Rx}}_{1} & {\text{Rx}}_{2} & \cdots {\text{Rx}}_{n}\\ \left|\;\right. & \left|\;\right. & \left|\;\right. \end{array}\right]}^{3\times n}=\left[\begin{array}{cccc} w_{1}y_{1}^{T}{\text{Rx}}_{1} & \; & \; & *\\ \; & w_{2}y_{2}^{T}{\text{Rx}}_{2} & \; & \;\\ \; & \; & \ddots & \;\\ {}* & \; & \; & w_{n}y_{n}^{T}{\text{Rx}}_{n} \end{array}\right]. \end{array}$$

Therefore,

(27) $$\begin{array}{c} \overset{n}{\underset{i=1}{\sum }}w_{i}{y_{i}}^{T}{\text{Rx}}_{i}=\text{tr}\left({\text{WY}}^{T}\text{RX}\right)=\underset{\text{tr}\left(\text{AB}\right)=\text{tr}\left(\text{BA}\right)}{\underbrace{\text{tr}{\left(\text{RXWY}\right)}^{T}}}. \end{array}$$

We set *S* = XWY^*T*^. *S* is a real symmetric matrix, and *S*_SVD_ = *U*∑*V*^*T*^, where *U* and *V* are unit orthogonal matrices, that is, the result of Schmidt orthogonalization of the matrix composed of point cloud eigenvectors. When it is brought into formula (27), we get

(28) $$\begin{array}{c} \text{tr}\left({\text{RXWY}}^{T}\right)=\text{tr}\left(\text{RS}\right)=\text{tr}\left(\text{RU}\sum V^{T}\right)=\text{tr}\left(\sum V^{T}\text{RU}\right). \end{array}$$

Because *M* = *V*^*T*^RU, *V*^*T*^, *R*, and *U* are all unit orthogonal matrices, then *M* is also a unit orthogonal matrix and MM^*T*^ = 1; that is, the inner product of each row and column in *M* is 1. If *m* is assumed to be a column vector of *M*, then *m*_*j*_^*T*^*m*_*j*_ = ∑_*i*_*m*_ij_^2^ = 1 and there is

(29) $$\begin{array}{c} \text{tr}\left(\sum M\right)=\left(\begin{array}{cccc} \sigma_{1} & \; & \; & \;\\ \; & \sigma_{2} & \; & \;\\ \; & \; & \ddots & \;\\ \; & \; & \; & \sigma_{n} \end{array}\right)\left(\begin{array}{c} m_{11}m_{12}\cdots m_{1n}\\ m_{21}m_{22}\cdots m_{2n}\\ \vdots \\ m_{n1}m_{n2}\cdots m_{nn} \end{array}\right)=\overset{n}{\underset{i=1}{\sum }}\sigma_{i}m_{ii}\leq \overset{n}{\underset{i=1}{\sum }}\sigma_{i}. \end{array}$$

When *M* = *I*, tr(∑*M*) can take the maximum value, then

(30) $$\begin{array}{c} I=M=V^{T}\text{RU}\Rightarrow \;V=\text{RU}\Rightarrow \;R={\text{VU}}^{T}. \end{array}$$

From formula (30), it can be known that the rotation matrix is related to the eigenvectors of the point cloud. According to formula (30), the rotation matrix required for the registration of any two point clouds can be obtained. The above derivation process can help to understand the whole process of the ICP algorithm and lay the foundation for the subsequent improvement of the method.

## 3. Recognition of Student Weariness Emotion in English Classroom Based on Internet of Things and Big Data Technology

Figure 6 shows an example image of student weariness expression recognition in intelligent English classroom obtained with the support of the second part of the algorithm in this paper. Moreover, this paper uses the human skeleton model to locate human facial expressions and extracts the features of human facial expressions after locating the human facial expressions, so as to improve the recognition effect of human expressions.

Based on the summary of the theoretical framework of smarter classrooms, this research proposes a system model of smarter classrooms based on the Internet of Things and big data technology, as shown in Figure 7.

If students are very interested in a learning activity, they will take the initiative to pay attention to the learning activity, actively participate in the classroom learning activities, and maintain a high sense of pleasure. Based on the analysis of the explicit behavioral characteristics of students' interest and the characteristics of the smarter classroom environment and the research purpose of this study, this paper constructs a conceptual model of students' interest in classroom learning, as shown in Figure 8.

After constructing the students' weariness emotion recognition model in English classroom, the simulation model of this paper is carried out through the simulation model, and the students' expressions are recognized.  Figure 9 is an example image of facial expression recognition for students in English class.

After that, this paper verifies the effect of the student weariness emotion recognition system proposed in this paper, and the statistical weariness emotion recognition effect is shown in Table 1.

From the above test results, it can be seen that the student weariness emotion recognition system proposed in this paper can effectively identify students' weariness emotion, which has certain reference significance for teachers to adjust teaching in a timely manner and has a certain auxiliary effect on students' psychological counseling.

## 4. Conclusion

The school's mental health education mostly relies on mental health classrooms to pass on mental health knowledge; through case counseling, it solves psychological problems such as adolescents' psychological confusion and emotional disorders. In addition, various mental health activities such as psychological squares, psychological group assistance, psychological lectures, and psychological salons are carried out. However, in addition to school, the living environment of young people is also a large part of family and society, and even the Internet has become an important part of their lives. However, family participation is insufficient, community resources are limited, and the coverage of mental health preventive interventions is small. This paper combines intelligent Internet of Things technology and big data technology to construct an improvement model of students' weariness in English classrooms and promote the construction of mental health of students in English classrooms in colleges and universities. From the test results, it can be seen that the student weariness emotion recognition system in English classroom proposed in this paper can effectively identify students' weariness emotion.

## Figures and Tables

**Figure 1:** Schematic diagram of the registration principle based on covariance matrix.

**Figure 2:** The iterative process of Newton's method for solving equations.

**Figure 3:** Schematic diagram of the relationship between PFH points.

**Figure 4:** 3D local coordinate system.

**Figure 5:** Schematic diagram of FPFH weight relationship.

**Figure 6:** An example of student weariness emotion recognition in English classroom based on Internet of Things and big data technology.

**Figure 7:** Smart classroom system model based on Internet of Things and big data technology.

**Figure 8:** The recognition model of students' interest in English classroom learning.

**Figure 9:** Example image of facial expression recognition of students in English class.

**Table 1:** The recognition effect of the system proposed in this paper for weariness emotion.

Number	Expression recognition	Number	Expression recognition	Number	Expression recognition
1	86.44	17	85.21	33	89.89
2	82.56	18	80.60	34	79.71
3	81.46	19	79.32	35	81.86
4	87.52	20	89.18	36	81.95
5	85.86	21	89.64	37	88.37
6	84.82	22	81.33	38	88.63
7	84.65	23	86.65	39	80.45
8	88.08	24	87.41	40	82.67
9	81.34	25	83.96	41	81.69
10	79.32	26	80.82	42	89.49
11	86.94	27	87.48	43	83.00
12	79.82	28	83.29	44	90.88
13	87.49	29	82.63	45	82.53
14	84.75	30	80.22	46	85.35
15	88.15	31	83.17	47	81.45
16	88.39	32	85.34	48	85.74

## Data Availability

The data used to support the findings of this study are available from the corresponding author upon request.
